RETRACTED

# The Significance of Apolipoprotein-A in the Long-Term Death of Patients with STEMI

**DOI:** 10.1155/2022/5941117

**Published:** 2022-01-15

**Authors:** Guoli Lin, Wen Chen, Caizhi Dai, Kaizu Xu

**Affiliations:** Department of Cardiology, The Affiliated Hospital of Putian University, Putian University, Putian, Fujian, China

## Abstract

**Objective:**

To analyze apolipoprotein-A for its predictive value for long-term death in individuals suffering from acute ST-segment elevation myocardial infarction following percutaneous coronary intervention.

**Methods:**

We selected patients suffering from acute ST-segment elevation myocardial infarction who underwent emergency PCI at the Affiliated Hospital of Putian University from January 2017 to August 2019. The patients were divided into a high-Apo-A group and low-Apo-A group, and we observed all-cause deaths of patients in the 2 groups within 2 years.

**Results:**

The ROC curve analysis indicated the best critical value for predicting 2-year mortality as 0.8150 (area under the curve was 0.626, sensitivity 75.1%, and specificity 51.9%). There was no statistical difference among the two groups in gender, age, lesion vessel, and comorbidities. The two groups had statistically significant differences in apolipoprotein-B/A, high-density lipoprotein, apolipoprotein-A, and hypersensitivity C-reactive protein. Correlation analysis showed a significant negative correlation between apolipoprotein-A and hypersensitive C-reactive protein. The results of the 24-month analysis indicated the incidence of all-cause mortality as higher in the low-Apo-A group, and Kaplan–Meier survival analysis showed the same trend.

**Conclusion:**

Apolipoprotein-A can predict the potential for long-term mortality among individuals having acute ST-segment elevation myocardial infarction.

## 1. Introduction

Over the past half a century, the global prevalence of coronary atherosclerotic heart ailment has grown rapidly. Acute ST-segment elevation myocardial infarction (STEMI) entails a critical type of heart ailment, which is the primary cause of mortality. After decades of standardized prevention in developed countries, the incidence of STEMI has decreased significantly, while China has shown a trend of rapid growth. In the ten years leading up to 2011, the rates of admission among STEMI patients have grown by almost 4 times in China (male patients increased from 4.6/100000 to 18/100000; female patients increased from 1.9/100000 to 8/100000). From 2013, the fatality rate in cases of acute myocardial infarction across nonurban locations has been high compared to that of urban locations.

Elevated concentration of low-density lipoprotein cholesterol as well as reduced concentration of high-density lipoprotein cholesterol can elevate the danger of atherosclerotic cardiovascular diseases [1]. Low-density lipoprotein particles are produced by significantly low-density lipoprotein in distribution, which are necessary in the transfer of cholesterol to peripheral tissue from the liver. In contrast, high-density lipoprotein particles have a major role in the reverse transfer of cholesterol to the liver from peripheral tissue [2]. The composition of low-density lipoprotein particles includes an apolipoprotein-B (Apo-B) molecule; thus, the number of Apo-B molecules is equal to that of extra-low-density lipoprotein. It is also equal to extra-low-density lipoprotein-derived elements in distribution [3]. Apolipoprotein-A is a primary component of high-density lipoprotein. Even though each high-density lipoprotein element could contain up to 5 apolipoprotein-A molecules, systematic apolipoprotein-A levels may indicate high-density lipoprotein cholesterol concentration, and Apo-A is not dependent on high-density lipoprotein cholesterol in predicting cardiovascular ailment risk. Some experiments have shown that, in untreated and statin-treated people, Apo-B, Apo-A, and their ratio (Apo-B/A) are identified as higher than low-density lipoprotein cholesterol. In turn, high-density lipoprotein cholesterol can more accurately predict the factors of cardiovascular disease [4]. Some studies have shown that apolipoprotein and non-high-density cholesterol are at least as powerful as classic indicators such as low-density cholesterol and sum cholesterol in predicting the occurrence of acute myocardial infarction [5]. However, only a few studies exist on its correlation and risks of long-term death in people with STEMI after PCI. The aim of the current study was to elucidate the predictive value of apolipoprotein-A in long-term mortality following percutaneous coronary medication in individuals with acute ST-segment elevation myocardial infarction, so as to guide the prognosis of STEMI patients after PCI.

RETRACTED

## 2. Methodology and Materials

### 2.1. Study Design and Populations

This research was reviewed and permitted by the Affiliated Hospital of Putian University Hospital Review Board.

200 individuals with acute ST-segment elevation myocardial infarction and who underwent emergency PCI at the Affiliated Hospital of Putian University were identified for participation. The determination of the disease conforms to the steps for the identification and management of the disease as stipulated in 2015 by the Chinese Medical Association [6]. The exclusion criteria are based on the following conditions: chronic inflammatory diseases, accompanied by active infection, malignant tumors, kidney and liver failure, and autoimmune and hematological diseases.

### 2.2. Data Collection

All patients' basic clinical data and laboratory examination results, as well as PCI information, were gathered. All information was selected from the hospital's digital medical record system as well as the PCI record. Also, angiographic outcomes were analyzed through quantitative coronary artery measurement, with the mode of PCI operation being determined by highly competent operators. Still, data used in this study come from the Affiliated Hospital of Putian College based on the help of its information center and the intervention catheterization rooms.

### 2.3. Group

According to Apo-A's critical value used in the prediction of 24-month all-cause death in the subject working characteristic curve (receiver operating characteristic curve, ROC), the individuals were categorized into high-Apo-A and low-Apo-A groups.

### 2.4. Follow-Up

Upon completing the PCI, follow-up on the patients was conducted throughout their hospitalization. This was achieved at the end of one month, six months, twelve months, eighteen months, and twenty four months, respectively. In achieving the follow-up process, the researchers used telephone and outpatient follow-up as well as noting of death and cessation of the process upon death.

### 2.5. Statistical Analysis

The choice of statistical analysis software for this study was the Statistical Package for Social Sciences software (SPSS 23.0 developed for Windows by IBM from USA). The process entailed expressing the measurement data in consistence with normal distribution by *x* ± *s*. The independent sample *t*-test is then selected to facilitate group comparisons as defined in the study. The data that were counted were also expressed as an example (%), and the comparison between groups was achieved through the chi-square test. The study also used the ROC curve in evaluating the predictive value of Apo-A in predicting all-cause deaths. The survival curve was estimated and drawn using the method stipulated by Kaplan–Meier, with the variance between the two groups of curves being compared using the method of log rank. The difference was statistically significant with a value of less than 0.05).

## 3. Findings

### 3.1. Patients' Baseline Traits

The study included 200 patients, with an age of (63.93 ± 11.59) years, of which 84.0% were males. The results of ROC curve portrayed that the ideal critical value in the prediction of 24-month death rate was 0.8150 (area under the curve was 0.626, sensitivity 75.1%, and specificity 51.9%, Figure 1). Based on this, participants were grouped into a high-Apo-A (Apo-A ≥ 0.8150) group and low-Apo-A (Apo-A < 0.8150) group.

RETRACTED

### 3.2. Comparing General Clinical Data across the Groups

In the high-Apo-A group, 118 males as well as 25 females were recorded, and the average age for the group was 64.43 ± 11.35 years, including 51 with hypertension and 31 with diabetes. In the low-Apo-A group, 50 males as well as 7 females were recorded with average age being 62.67 ± 12.17 years, including 16 with hypertension and 15 with diabetes. The study did not find a significant variance in age, culprit vessels, sex, complication, heart rate, diastolic and systolic blood pressures, and hospitalization days across the identified categories (see Table 1).

### 3.3. Comparison of the Two Groups for Tests from Laboratory

The study did not record any significance in terms of the variance in neutrophil count, white blood cell count, hemoglobin, triglyceride, serum creatinine, serum uric acid, D-dimer, troponin, B-type N-terminal natriuretic peptide, hypersensitive thyrotropin, glycosylated hemoglobin, and ejection fraction across the two categories (*p* > 0.05). However, high-density lipoprotein, apolipoprotein-A, hypersensitive C-reactive protein, and apolipoprotein-B/A across the two categories portrayed significant differences (*p* < 0.01). See Table 2 for the specific values.

### 3.4. Correlation Analysis

In bivariate correlation analysis, the study found a negative and significant correlation pitting apolipoprotein-A against hypersensitive C-reactive protein (*r* = −0.238, *p* < 0.001, see Figure 2).

### 3.5. Comparison of Clinical Prognosis across the Two Categories

The findings for the 2-year follow-up showed that compared with the high-Apo-A group, the low-Apo-A group had a higher incidence of all-cause mortality (*p* value <0.05) (see Table 3). The same trend was observed in the results of the survival analysis by Kaplan–Meier (Figure 3).

## 4. Discussion

Apolipoprotein-A is the main apolipoprotein in high-density lipoprotein. Its function is to transfer cholesterol into the liver from the body tissue, thus facilitating catabolism. Still, the lipoprotein inhibits the depositing of cholesterol in the walls of the blood vessels. Therefore, apolipoprotein-A can inhibit the formation of atherosclerotic plaque. In contrast, apolipoprotein-B is the primary apolipoprotein in low-density lipoprotein. Low-density lipoprotein cholesterol is a significant constituent in atherosclerotic plaque, thus making it the main risk factor of atherosclerosis [7].

In a retrospective study of 32100 people, it was observed that apolipoprotein-B levels increased and apolipoprotein-A levels decreased in individuals diagnosed with acute myocardial infarction. Apolipoprotein-A and apolipoprotein-B have better discrimination ability than low-density and high-density lipoproteins [8]. In past studies, apolipoprotein-B and non-high-density cholesterol have been found at least as powerful as more classic indicators such as low-density and total cholesterol in predicting the development of acute myocardial infarction. Similar results were observed even in individuals with statin treatment. AMORIS and INTERHEART studies also confirmed that apolipoprotein-A and apolipoprotein-B are closely related to acute myocardial infarction [6]. The proportion of plasma apolipoprotein-B/A can indirectly showcase the balance among antiatherosclerotic factor as well as proatherosclerotic factor. The higher the ratio of apolipoprotein-B/apolipoprotein-A, the more the cholesterol in plasma. The cholesterol has a higher probability of being deposited along the walls of the artery. The lower the apolipoprotein-B/apolipoprotein-A ratio, the greater the reverse transport and other beneficial functions. In this study, the ratio of apolipoprotein-B/apolipoprotein-A was lower in the high-Apo-A group, which was consistent with the abovementioned conclusion.

RETRACTED

As an inflammation marker, the C-reactive protein which has a high sensitivity is a powerful indicator of future cardiovascular incidents. Some prospective cohort analyses have proved a positive association between higher concentrations of hypersensitive C-reactive protein and an increased probability of cardiovascular ailment, and it is an important marker of inflammatory injury in people diagnosed with acute myocardial infarction [9]. Through the inflammation process, the proportion of triglyceride, phospholipid, and cholesterol in low-density lipoprotein, low-density lipoprotein, and very-low-density lipoprotein particles increased, while the proportion of cholesterol and triglyceride in high-density lipoprotein particles decreased [10]. In this study, the value of hypersensitive C-reactive protein in the low-Apo-A category was higher compared to that of the high-Apo-A group, and there was a negative correlation between Apo-A and hypersensitive C-reactive protein, suggesting that Apo-A can inhibit inflammation and improve the management of individuals that have acute myocardial infarction. The possible mechanisms may be as follows: recombinant Apo-A increases the ability of HDL efflux and reduces atherosclerosis; Apo-A determination is the key decisive factor of macrophage cholesterol efflux ability, and Apo-A protein can reduce atherosclerosis by regulating macrophage cholesterol efflux. Other studies have shown that individuals having acute coronary syndrome as well as those with stable atherosclerotic disease were injected with remodeled insoluble human Apo-A preparation (CSL112), which confirmed increased acute cholesterol outflow function in both populations, and CSL112 reduced major adverse cardiovascular events [11]. In this study, it was found that the AUC value of apolipoprotein-A for predicting all-cause death of acute STEM infarction is 0.626, apolipoprotein-A of 0.8150 g/L can be used as the best critical value of overall mortality in acute STEM infarction, and its specificity sensitivity levels were 0.51 and 0.75, respectively. When Apo-A <0.8150 g/L, individuals that have acute ST-segment elevation myocardial infarction are likely to lead to poor clinical results, which should arouse the vigilance of clinicians.

RETRACTED

## 5. Conclusions

APO-A can well distinguish the danger of STEMI in emergency PCI individuals that have acute ST-segment elevation myocardial infarction. Increased Apo-A can reduce the likelihood of mortality in people that have STEMI. Therefore, it is recommended that Apo-A be used in the assessment of risks for PCI patients that have been diagnosed with acute myocardial infarction.

This study faces a number of limitations. In particular, the study is limited in the choice of Apo-A in the complete set of biochemistry at the time of hospitalization as the observation index, there is absence of comparison, and it may be better to be able to measure Apo-A multiple times for a comparative study; secondly, the 2-year follow-up time of this study is shorter, which may affect the observation of the long-term prognosis of the two groups of patients. Still, the current study is not characterized by a randomized control, thus missing out on the opportunity of evaluating the predictive value of Apo-A on the mortality of individuals with STEMI after PCI.

## Figures and Tables

**Figure 1:** The receiver operating characteristic curve of Apo-A predicting 2-year all-cause death in individuals with STEM disease.

**Figure 2:** Representation of the correlation between apolipoprotein-A and hypersensitive C-reactive protein.

**Figure 3:** Kaplan–Meier survival curve of 2-year all-cause death in the high-Apo-A group and low-Apo-A group.

**Table 1:** Comparing basic data of the groups of patients.

Variable	High-Apo-A group	Low-Apo-A group	*p* value
Number of cases	143	57	—
Age (years)	64.43 ± 11.35	62.67 ± 12.17	0.334
Male (%)	118 (82.50)	50 (87.70)	0.403
Hypertension (%)	51 (35.70)	16 (28.10)	0.325
Diabetes (%)	31 (21.70)	15 (26.30)	0.577
LM (%)	4 (2.80)	0 (0)	0.258
LAD (%)	60 (55.9)	28 (48.10)	0.433
LCX (%)	15 (10.50)	2 (3.50)	0.160
RCA (%)	44 (30.80)	26 (45.60)	0.136
Heart rate (beats/min)	75.85 ± 16.90	80.74 ± 17.04	0.070
SBP (mmHg)	126.85 ± 24.29	119.42 ± 26.90	0.073
DBP (mmHg)	77.79 ± 15.80	75.79 ± 16.96	0.490
Hospitalization days	9.42 ± 4.13	10.25 ± 5.23	0.252

LAD, left anterior descending artery; DBP, diastolic blood pressure, RCA, right coronary artery; LCX, left circumflex artery; SBP, systolic blood pressure; LM, left main coronary artery.

RETRACTED

**Table 2:** Comparative analysis of the two categories of laboratory results.

Variable	High-Apo-A group	Low-Apo-A group	*p* value
Number of cases	143	57	—
WBC count (10^9^/L)	11.30 ± 4.35	12.68 ± 7.28	0.184
Hemoglobin (g/L)	138.52 ± 16.48	135.85 ± 22.20	0.351
Neutrophil count (10^9^/L)	9.17 ± 4.57	9.33 ± 4.48	0.819
Apolipoprotein-A (g/L)	0.99 ± 0.13	0.70 ± 0.72	0.001
Apolipoprotein -B/A	0.95 ± 0.32	1.12 ± 0.43	0.003
Triglycerides (mmol/L)	1.66 ± 0.66	1.84 ± 3.24	0.621
High-density lipoprotein (mmol/L)	1.12 ± 0.28	0.86 ± 0.14	0.001
Serum creatinine (umol/L)	75.77 ± 19.47	77.32 ± 32.04	0.888
Serum uric acid (umol/L)	377.33 ± 97.62	368.47 ± 110.35	0.121
D-dimer (ug/mL)	0.81 ± 1.44	1.56 ± 5.56	0.094
High-sensitivity C-reactive protein (mg/L)	8.56 ± 16.52	21.52 ± 34.97	0.001
Troponin I (ng/ml)	33.53 ± 32.84	35.02 ± 33.30	0.773
NT-pro-BNP (Pg/ml)	1509.55 ± 3940.31	1165.89 ± 1701.20	0.528
Hypersensitivity thyrotropin (uIU/ml)	1.28 ± 1.41	1.14 ± 0.65	0.601
Glycated hemoglobin (%)	7.18 ± 1.76	7.24 ± 2.30	0.862
Ejection fraction (%)	58.210 ± 7.82	58.44 ± 7.90	0.859

WBC, white blood cell; NT-pro-BNP, N-terminal pro-B-type natriuretic peptide.

**Table 3:** Follow-up results of clinical prognosis for 2 years in the high-Apo-A group and low-Apo-A group (case (%)).

Group	Number of cases	All deaths
High-Apo-A group	143	13 (9.10)
Low-Apo-A group	57	14 (24.60)
*X* ^2^	—	8.353
*p* value	—	0.006

## Data Availability

The simulation experiment data used to support the findings of this study are available from the corresponding author upon request.
